# In Vitro Antibacterial Potential against Multidrug-Resistant *Salmonella*, Cytotoxicity, and Acute Biochemical Effects in Mice of *Annona muricata* Leaf Extracts

**DOI:** 10.1155/2022/3144684

**Published:** 2022-08-16

**Authors:** Moses Njutain Ngemenya, Rodolph Asongana, Denis Zofou, Rita Ayuk Ndip, Lamson Ottotoh Itoe, Smith Borakaeyabe Babiaka

**Affiliations:** ^1^Department of Biochemistry and Molecular Biology, University of Buea, P.O. Box 63, Buea, Cameroon; ^2^Department of Medical Laboratory Sciences, University of Buea, P.O. Box 63, Buea, Cameroon; ^3^Department of Chemistry, University of Buea, P.O. Box 63, Buea, Cameroon

## Abstract

The treatment of *Salmonella* infections is threatened by multidrug resistance necessitating the search for alternative treatments, such as from medicinal plants. There are several reports on the antibacterial activity of *Annona muricata*. This study assessed the activity against multidrug-resistant (MDR) *Salmonella* and also the toxicity of the leaves of this plant. The hexane and methanol extracts of the leaves were screened against characterized MDR isolates by disc diffusion and microdilution methods. A cytotoxicity test was performed on monkey kidney epithelial cells; an acute toxicity test was conducted in BALB/*c* mice and the liver and kidney functions were assessed at the end of the test. Both extracts recorded weak activity in the disc test. Conversely, the extracts showed a wide range of activity against specific *Salmonella* isolates in the microdilution assay, and the lowest minimum inhibitory concentration value recorded was 0.0625 mg/mL. The hexane extract (ANO_HEX_) was not cytotoxic (CC_50_ = 57.7 *µ*g/mL) and was also not toxic to the mice at 2000 mg/Kg bodyweight, while the methanol extract (ANO_MET_) was cytotoxic (CC_50_ = 18.44 *µ*g/mL), and mortality was recorded at 2000 mg/Kg but not at 300 mg/Kg. There were no significant changes in biomarkers of the liver (alanine aminotransferase and aspartate aminotransferase) and kidney (creatinine and urea) functions (*P* > 0.05), except for ANO_HEX_ which significantly decreased creatinine (*P* = 0.01), in the test mice which was not considered a toxic effect. In conclusion, this study has demonstrated high bacteriostatic activity against MDR *Salmonella* and a low risk of toxicity of *A. muricata* leaves. Hence, the leaves are a potential alternative treatment for resistant *Salmonella* infection. The natural products should be further investigated in vitro and in vivo.

## 1. Introduction

The global burden of *Salmonella* infections, both typhoidal and nontyphoidal, is high alongside a high mortality rate [1]. The prevalence is higher in Africa largely due to poor water and food hygiene. In the past, these infections were successfully controlled with the use of antibiotics and improved water quality [2]. Presently, these infections persist in poor settings due to the emergence of multidrug-resistant (MDR) clades of *Salmonella*. Resistance first emerged to the first-line antibiotics, which are ampicillin, trimethoprim-sulfamethoxazole, and chloramphenicol, and later to tetracycline and streptomycin. This led to the adoption of fluoroquinolones and cephalosporins which were effective in the treatment of infections with MDR strains [2]. However, recent evidence shows a significant increase in antibiotic resistance with an increase in nonsusceptibility to ciprofloxacin in the United States [3, 4]. Studies have reported increasing resistance of *S. typhi* to ceftriaxone and azithromycin in India [5] and increasing MDR strains in Africa [6]. A recent study in Southwest Cameroon detected MDR strains with multiple resistant genes and considerable resistance to ciprofloxacin [7].

The resistance challenge posed by *Salmonella* has led to a multifaceted approach to counter this threat which includes antibiotic stewardship, discovery and development of new efficacious antibacterials from medicinal chemistry, and research on alternative medicines from natural sources among other approaches [8, 9]. A natural source of interest is *Annona muricata* (Annonaceae), a fruit tree known in Cameroon as soursop, which is widely distributed in tropical and subtropical regions of the world [10]. In ethnomedicine, the decoctions of the bark, root, seed, and leaf are widely used in various applications. The fruit is used in the treatment of diarrhoea, dysentery, and parasitic infections among others. The leaves are used to treat skin ailments, pain, hypertension, diabetes, and respiratory system diseases including asthma, malaria, and cancer [11]. The leaves are used to treat typhoid fever in Cameroon [12]. In vitro studies have revealed a wide range of pharmacological properties of the leaves which include antiproliferative activity against some cancer cell lines, promising antiparasitic activities, antioxidants, and also insecticidal properties [11]. In vivo studies of the leaf extracts have revealed antihypertensive, hypoglycaemic, anticancer, hepatoprotective, and wound healing properties. Over two hundred phytochemicals have been isolated from the leaves and other parts of this plant and structurally characterized. They include mostly acetogenins, alkaloids, and phenols and the biological activities of some of them have been reported [11].

A few in vitro studies have demonstrated antibacterial activity of the leaf extracts but have been largely limited in scope [13, 14] and not extensive. These studies were performed on very few species [15]. In particular, studies against MDR bacteria are very rare. The aqueous leaf extract showed moderate inhibition of a MDR *Mycobacterium* strain [16]. The mechanisms of action of the leaf extracts have not been elucidated but are thought to include inhibition of nucleic acid synthesis and some enzymes [11]. The aqueous leaf extract potentiated the activity of some antibiotics against methicillin-resistant *Staphylococcus aureus* [17]. Considering the well-documented use of this plant in the treatment of infectious diseases and the limited reports on its antibacterial activity, this study aimed to investigate the activity of extracts of *A. muricata* leaves against MDR clinical *Salmonella* isolates and also the cytotoxicity and acute toxicity in mice.

## 2. Materials and Methods

### 2.1. Plant Collection and Preparation of Extracts

The leaves of *A. muricata* were collected in Buea, and a voucher specimen was prepared and authenticated by Mr. Peter Njimba at the Limbe Biodiversity and Conservation Centre, Cameroon, and was assigned voucher specimen number SCA12826. The crude extracts were prepared as described [18]. Briefly, the leaves were dried under shade for three weeks and ground to a fine powder using a grinding mill (CE SGS ISO9001, China). The powder was weighed, macerated separately in hexane and methanol each for 72 h, and then filtered using Whatman filter paper no.1. The filtrate was concentrated by rotary evaporation (BUCHI Rotavapor R-200, Switzerland) at 65°C (hexane) and 80°C (methanol). Each crude extract was dried and then weighed and stored at 4°C in a refrigerator until use.

### 2.2. Sources of Bacteria

The test bacteria were sixteen MDR clinical isolates of *Salmonella* from specimens of patients obtained from four medical laboratories in the South West region of Cameroon. They were characterized using cultural, biochemical, and molecular techniques and were reported in a recent study [7]. The isolates comprised of four *S. typhimurium*, eight *S. typhi*, and four *S. paratyphi*. Two control strains used were *Salmonella typhimurium* (ATCC14028) and *Salmonella enteriditis* (ATCC13076), obtained from the American Type Culture Collection, Manassas, Virginia, United States of America.

### 2.3. Anti-*Salmonella* Screens

A 25 mg/mL stock solution of the hexane extract was prepared by dissolving 25 mg of the extract in 60 *µ*L of acetone, and 940 *µ*L of distilled water added and mixed by vortexing. A stock solution of the methanol extract was prepared similarly by dissolving 25 mg in 250 *µ*L of 2% dimethyl sulfoxide (DMSO) (SIGMA, Burlington, USA), and 750 *µ*L of distilled water was added. Mueller–Hinton (MH) agar and broth (Liofilchem, Italy) were prepared according to the manufacturer's instructions.

#### 2.3.1. Antibacterial Screen by Disc Diffusion

The anti-*Salmonella* activity was determined by disc diffusion as described [18, 19]. In brief, a McFarland 0.5 bacterial suspension (1.5 × 10^8^ CFUs/mL) was prepared and spread on a MH agar plate. Sterile discs prepared from Whatman filter paper were placed on the agar surface, and 10 *µ*L of extract solution containing 1 mg of extract was added onto the disc. This was allowed to dry for 30 minutes and then incubated at 37°C (DHP-9052, England) for 24 hours, after which the diameters of zones of inhibition were measured manually using a millimetre ruler [20].

#### 2.3.2. Antibacterial Screen by Microdilution

The minimum inhibitory concentration (MIC) was determined as previously described [19], with some modifications in volumes used. In brief, extract stock solutions (ANO_Hex_ and ANO_Met_) were prepared by dissolving 40 mg of each crude extract in 200 *µ*L of DMSO and 800 *µ*L of MH broth added and mixed thoroughly by vortexing. Bacterial suspensions (McFarland 0.5) were prepared and further diluted 1 : 150 with MH broth to approximately 1 × 10^6^ CFUs/mL. Extract solution (75 *µ*L) was added to the required wells in the 96-well microtitre plate in duplicate followed by 75 *µ*L of bacterial suspension giving final extract concentrations of 0.0625, 0.125, 0.25, 0.5, 1, 2, 4, 6, 8, and10 mg/mL containing 5 × 10^5^ CFUs/mL of *Salmonella* cells. The baseline optical densities (OD) of the wells were read at 595 nm (Emax microplate reader, Molecular Devices, San Jose, USA) and incubated at 37°C (DHP-9052, England) for 24 h. The plates were visually observed for inhibition and OD reread. The change (∆) in OD was determined and percentage inhibitions of bacterial growth were calculated using the following formula:

(1) $$\begin{array}{c} \%\text{ inhibition}=\frac{\Delta \text{OD negative control}-\Delta \text{OD extract}}{\Delta \text{OD negative control}}\times 100. \end{array}$$

The MIC was taken as the lowest concentration which showed >50% inhibition of bacterial growth. To determine the minimum bactericidal concentration (MBC), the contents of all MIC wells devoid of bacterial growth were mixed and 10 *µ*L of each was spotted on agar, incubated at 37°C for 24 h and observed for growth (CFUs). The MBC was recorded as the lowest concentration of the corresponding spot without growth.

### 2.4. Toxicity Tests

#### 2.4.1. Cytotoxicity Test

The cytotoxicity test was done as described by Ngemenya et al [18], where a detailed description is outlined. Briefly, monkey kidney epithelial cells were cultured to confluence in a complete culture medium (RPMI 1640 containing newborn calf serum) at 37°C in 5% CO_2_ humidified air. The medium was discarded; the cells were washed with incomplete medium (no calf serum), dislodged with trypsin, centrifuged, and the incomplete medium replaced followed by counting of the cells. The cells were seeded in a 96-well microtitre plate (3000 cells/100 *µ*L) and cultured as above. When the cells were confluent, the extract was added (100 *µ*L) at final concentrations from 15 to 1000 *μ*g/mL. Positive (30 *μ*M auranofin) and negative (2% DMSO in complete culture medium) controls were included, and the plate was incubated as above for 5 days. Then, the medium was discarded, the incomplete medium was added, and the plate decolourised in a shaker. Then, 100 *µ*L of MTT (5 mg/mL) was added and incubated for 30 mins, and the formazan dissolved by adding 100 *µ*L DMSO. The ODs were read at 595 nm, and percentage inhibition of cell growth was calculated relative to the negative control as described [18].

#### 2.4.2. Acute Toxicity Test

This study was approved by the Institutional Animal Care and Use Committee (reference number: UB-IACUC N^0^ 08/2020) and was performed as described with some modifications [21, 22] and in accordance with guidelines of the Organization for Economic Cooperation and Development version 423 [23]. In brief, two groups (control and test) of five nine-week-old adult BALB/*c* mice (two females and three males) were obtained from the animal house of the laboratory, and the experiment was conducted in an adjacent room. One animal from the test group was weighed, fasted (with water), and administered an extract dose of 2000 mg/kg bodyweight by oral gavage; it was fasted further for 2 hours and provided food and then observed as described [21]. Following the survival of the treated animal, the other four were fasted and treated the same. In case the single animal that was fasted and treated died, the test was repeated at 300 mg/kg bodyweight as recommended [23]. All animals were monitored for signs of toxicity for 14 days, weighed, then fasted overnight, and anesthetized (intraperitoneal ketamine/xylazine, 90/10 mg/kg), and blood was collected by retro-orbital bleeding. The blood was coagulated (30 mins) and centrifuged (2200 rpm × 15, minutes Eppendorf centrifuge 5702 R), and biochemical tests were performed using the Chronolab kit (Switzerland) for alanine aminotransferase (ALT), aspartate aminotransferase (AST), urea, and Biorex diagnostic kit (United Kingdom) for creatinine, following manufacturer's instructions.

### 2.5. Phytochemical Analysis of Extracts

Phytochemical analyses were done to determine the chemical classes of secondary metabolites in each extract, using standard chemical tests as described [24, 25]. Tests were done for alkaloids, flavonoids, steroids, tannins, cardiac glycosides, saponins, and phenolics, and their relative abundances in each extract were determined.

### 2.6. Data and Statistical Analysis

The CC_50_ (concentration which kills 50% of cells) was determined from a plot of log concentration against percentage inhibition generated using GraphPad Prism 5.0 software (Graph Pad Prism INC., CA, USA). Data on biochemical markers were analysed using the same software. An unpaired two-tailed *t* test was used to compare parameters for control and test animals to determine any significant difference (*P* < 0.05).

## 3. Results

### 3.1. Antibacterial Activity of Crude Extracts

The hexane and methanol extracts (ANO_HEX_ and ANO_MET_, respectively) showed weak activity in the disc diffusion test against all the sixteen MDR *Salmonella* isolates and control strains, and the highest diameter of zone of inhibition was 8 mm. The positive control (ciprofloxacin) was very effective and produced inhibition zones in the range of 25–37 mm, while the negative control produced no zone of inhibition. In the microdilution assay, the two extracts showed MIC values ranging from 0.0625 to 8 mg/mL against individual MDR *Salmonella* isolates. The lowest MIC value corresponding to the highest activity was 0.0625 mg/mL and was produced by ANO_Hex_ and ANO_Met_ against three and four clinical isolates, respectively, out of a total of 16 tested isolates. The methanol extract recorded MICs in the high activity range (≤2 mg/mL), for 12 isolates as against 6 for the hexane extract; hence, the methanol extract had higher activity against the MDR isolates (Table 1). No MBC values were recorded for both extracts in the concentration range tested, suggesting the extracts were bacteriostatic.

### 3.2. Cytotoxicity of Extracts

The cytotoxicity test on monkey kidney epithelial cells revealed that the methanol extract, ANO_Met_, had a CC_50_ value of 18.44 *µ*g/mL which is lower than the cutoff point for lack of cytotoxicity (30 *µ*g/mL) [18]; this indicates that this extract is cytotoxic. The hexane extract, ANO_Hex_, recorded a CC_50_ value of 57.7 *µ*g/mL; hence, it was not cytotoxic. The relative selectivity was poor (obtained from the formula: CC_50_/MIC in *µ*g/mL), as seen from the very low selectivity index values of 0.92 and 0.29 for the hexane and methanol extract, respectively.

### 3.3. Acute Toxicity of Extracts

For the hexane extract of *A. muricata*, no sign of acute toxicity was observed and no death of mice was recorded at 2000 mg/kg bodyweight. There was no significant difference in bodyweights between the two groups of mice (*P*=0.7866). The methanol extract (ANO_MET_) was toxic at 2000 mg/kg; the animals were inactive and weak 2 hours postdosing and all the mice died between days 3 and 4. When the test was repeated at the lower recommended dose of 300 mg/Kg (OECD, 2001), no sign of acute toxicity and no mortality were recorded, suggesting the LD_50_ is below 2000 mg/Kg. The average body weights of the control group decreased by 2% while that of the test group increased by 5% resulting in a significant difference in bodyweights (*P*=0.0430).

### 3.4. Biochemical Effects on Liver and Kidney Functions

The hexane extract (at a nonlethal dose of 2000 mg/Kg) showed no significant difference between the control (2% DMSO) and test (ANO_Hex_) groups of mice for ALT, AST, and urea, with *P* values of 0.1752, 0.9633, and 0.8417, respectively. But creatinine decreased significantly in the test group (*P*=0.0113) as shown in Figures 1 and 2. The AST: ALT ratio was 2.7 suggesting adverse toxicity.

For the methanol extract (at a nonlethal dose of 300 mg/Kg), there was no significant difference between the control (2% DMSO) and test (ANo_Met_) groups of mice with *P* values of 0.2260, 0.7631, 0.9693, and 0.5370 for AST, ALT, urea, and creatinine, respectively, as shown in Figures 3 and 4. The AST : ALT ratio was 6.3 suggesting adverse toxicity.

### 3.5. Phytochemical Composition and Yield of Extracts

The hexane extract had a yield of 57.7% with relatively high amounts of tannins, saponins, and steroids and low amount of flavonoids, while the methanol extract had a relatively much lower yield of 8.8%, but the test revealed the presence of high amounts of steroids and flavonoids and low amounts of tannins, saponins, and phenolics. Alkaloids and cardiac glycosides were not detected in both extracts.

## 4. Discussion

In the context of the reported wide-ranging antimicrobial activity of *A. muricata*, the anti-*Salmonella* activity was investigated against MDR clinical isolates. The two extracts showed rather negligible activity in the disc test; however, in the microdilution assay, very high activity was recorded against some individual isolates. The weak activity in the disc test could be due to the presence of a low content of bioactive secondary metabolites in the amount of crude extract (1 mg) used. However, several factors are known to affect the diameter of the zone of inhibition of substances in the disc test which is based on the principle of the diffusion of compounds outward from the disc [27]. For plant extracts in particular, an important factor is the polarity of the compounds in the extracts which are largely nonpolar, hence diffuse slowly in agar which is an aqueous medium.

The methanol extract recorded high activity in the microdilution test (MIC ≤2 mg/mL) against most isolates than the hexane extract, indicating that it was more active against the MDR isolates. A dose-response relationship was observed in the activity of both extracts based on the MIC values; the higher the MIC value, the higher the cumulative number of isolates inhibited (Table 1). The wide range of the MIC values is probably due to variation in the magnitude of resistance as a consequence of the presence of different resistant genes in each *Salmonella* isolate as reported [7], resulting in varied susceptibility to the extracts. Some studies have been done on the antibacterial activity of *A. muricata*, but this is the first report on the activity of the leaf extract against MDR *Salmonella*. Most reported studies were limited in scope; whereby, aqueous extracts were investigated by the disc diffusion method only [13, 28], and studies involving MIC determination were mostly against two bacterial species, *Escherichia coli* and *Staphylococcus aureus* [14]. A study on the leaf ethanol extract reported MIC values of 2–4 mg/mL against *Salmonella* strains which were not characterized to establish whether they were resistant or not [12]. In another study, the aqueous leaf extract showed moderate inhibition of a MDR *Mycobacteriun* strain [16]. Both extracts in this study were not bactericidal in the concentration range tested (no MBC), suggesting they are bacteriostatic; their activity is likely due to the phytochemicals present in a high amount as mentioned above.

The low selectivity index values of the extracts are due to their low CC_50_ values which are close to the cutoff value for cytotoxicity (<30 *µ*g/mL) [18]. This reflects their potential to be toxic as seen with the methanol extract which was cytotoxic (low CC_50_ of 18.44 *µ*g/mL) and caused 100% mortality of mice at the relatively high dose of 2000 mg/Kg bodyweight, unlike the hexane extract. This suggests the toxic components are present in the methanol extract. No toxicity was recorded for the methanol extract at 300 mg/Kg indicating its toxicity is dose-dependent. Several other studies did not find cytotoxicity but recorded a wide-ranging degree of inhibition of many normal and cancer cell lines by different leaf extracts. The leaf ethanol extract strongly inhibited kidney epithelial cells (VERO, IC_50_ < 0.22 *µ*g/mL), while the hexane extract showed a moderate inhibition of human colon epithelial cells (CCD841, IC_50_ = 42.1 *µ*g/mL) [11].

All biochemical markers of toxicity were not significantly altered in test mice compared to control for both extracts. But the significant decrease in creatinine concentration in mice administered the hexane extract, suggests increased excretion of this waste product of metabolism, which does not imply kidney damage. However, the AST: ALT ratios were high for both extracts suggesting severe liver injury. Other studies have reported high AST: ALT ratios with significant histopathological changes in the liver tissue of treated animals, but no mortality was recorded suggesting possible reversible liver injury [29, 30].

There are some limitations to this study such as the relatively small number of MDR *Salmonella* isolates used in the test, and the results were not analysed according to the resistant genes in each isolate. Another limitation is that the natural products were not isolated and tested in order to identify the active ingredient in the extracts.

## 5. Conclusion

This study is the first to report the finding that *A. muricata* leaves possess high bacteriostatic activity against MDR *Salmonella*. It also showed a low risk of toxicity to mammals at relatively low doses. Hence, the leaves are potential alternative treatment for resistant *Salmonella* infections. The natural products in the leaves should be isolated and further investigated against MDR bacteria in vitro and in vivo.

## Figures and Tables

**Figure 1:** Effects of a single oral dose of 2000 mg/Kg hexane extract of *Annona muricata* leaves on mouse liver enzymes. The unpaired two-tailed *t-*test showed no significant difference between the control and test animals for ALT (alanine aminotransferase) (*P*=0.17) and AST (aspartate aminotransferase) (*P*=0. 96).

**Figure 2:** Effects of a single oral dose of 2000 mg/Kg hexane extract of *Annona muricata* leaves on mouse renal function biomarkers. The unpaired two-tailed *t-*test showed no significant difference for urea (*P*=0. 84) and a significant difference for creatinine (*P*=0. 01)^*∗*^ between the control and test animals.

**Figure 3:** Effects of a single oral dose of 300 mg/Kg methanol extract of *Annona muricata* leaves on mouse liver enzymes. The unpaired two-tailed *t-*test showed no significant difference between the control and test animals for ALT (alanine aminotransferase) (*P*=0.22) and AST (aspartate aminotransferase) (*P*=0. 96).

**Figure 4:** Effects of a single oral dose of 300 mg/Kg methanol extract of *Annona muricata* leaves on mouse renal function biomarkers. The unpaired two-tailed *t-*test showed no significant difference between the control and test animals for urea (*P*=0. 96) and creatinine (*P*=0. 53).

**Table 1:** Minimum inhibitory concentrations of *Annona muricata* leaf extracts against multidrug-resistant *Salmonella* isolates.

Extracts	MIC values (mg/mL)	No. of isolates^*∗*^	Cumulative no. of isolates	Activity
ANO_Hex_	0.0625	3	3	High
	0.125	2	5	
	2	1	6	
	4	3	9	Moderate
	6	1	10	
	8	6	16	Low

ANO_MET_	0.0625	4	4	High
	0.25	2	6	
	0.5	2	8	
	0.125	3	11	
	4	1	12	Moderate
	6	2	14	
	8	2	16	Low

Interpretation of MIC values (mg/mL): ≤2, high activity; >2 and <6, moderate activity; >6, low activity [26]. Extracts: ANO_Hex_ and ANO_Met_: hexane and methanol extracts of *A. muricata*, respectively. MICs, minimum inhibitory concentrations.

## Data Availability

The data used to support the findings of this study are available from the corresponding author upon request.
